This article has been retracted.

# The Curriculum Knowledge Analysis of Marxist Philosophy and System Theory Based on Association Rules

**DOI:** 10.1155/2022/4543851

**Published:** 2022-08-16

**Authors:** Yingli Pan

**Affiliations:** ^1^School of Philosophy and Government, Shaanxi Normal University, Xi'an 710062, China; ^2^Xi'an Peihua University, Xi'an 710125, China

## Abstract

Systems theory and Marxist philosophy are inextricably linked. Systems theory and Marxist philosophy are both methodologies in a sense and share the perspective of movement and development. The system theory is also embodied in the Marxist philosophy's conceptions of nature, social history, and epistemology. Studying the system theory in Marxist philosophy will undoubtedly benefit from having a solid understanding of the connection between system theory and that philosophy. It has become crucial to enhance the quality of instruction by analyzing student learning data and providing constructive criticism for teaching methods. The students' learning data from the course teaching Marxist philosophy and systems theory were mined and analyzed based on the Apriori algorithm, and strong association rules between the course teaching contents were generated. We can determine the challenging teaching material that has an impact on students' performance through the analysis of these generation rules, enabling teachers to use this feedback information to enhance their pedagogical approaches.

## 1. Introduction

System methodology includes the brand-new theoretical system known as system theory, which first appeared in the 1940s. System theory extracts various system theories and the common elements of these theories through the study of physics, mathematics, biology, chemistry, etc., in the natural sciences in order to achieve for research purposes [1] and to make abstract research objects more concrete. The philosophical idea it advances has a certain relationship to Marxist philosophy because everything exists in the system [2].

Data mining [3] is a popular technique for examining how well college students are learning. Data mining can analyze the factors that affect the students' performance, and the association rule algorithm [4] is one of the data mining. Simple mathematical statistics can only simply show the final learning effect of the students, and the potential information in the learning process has not been effectively analyzed. It is a crucial technique that can produce helpful feedback for the teaching process. The analysis of rules between courses is where the current association rule methods are most frequently used, as opposed to the analysis of rules between the various course contents. The key to determining whether a student passes a particular course is to look at the course's important and challenging material.

At present, association rules have been widely used in knowledge reasoning, analysis, and other work. By analyzing the connections between various knowledge points, knowledge connections can be mined [5, 6]. For example, literature [7] studies the application of association rules to the design of question answering systems; literature [8] studies some weakly supervised learning algorithms for association rules in large knowledge bases; literature [9] studies data mining technology and association of comprehensive application of rules; literature [10] studies methods to improve the quality of data association analysis. In addition to these studies on association analysis algorithms, more scholars have studied the application of association rule analysis in some specific fields, such as the application of association rules in English online mixed teaching [11], and the association rule model can be applied to students' thinking educational work [12]; Bi [13] studied the relationship between ideological and political teaching and mental health; Khan et al. [14] studied the impact of teaching on student performance based on data mining analysis; Chen [15] proposed that association rules are used in teaching evaluation work; some scholars use association rules in the scheduling and distribution of educational resources [16].

This paper uses the Apriori algorithm [17] to deeply mine and analyze the learning data of students of Marxist philosophy and systems theory, generate strong association rules between the teaching contents of the course, analyze the difficult content that affects the performance, according to the focus of the course syllabus content and analysis of the difficult content, put forward the improvement of the course teaching plan, and help improve the quality of students' learning and the quality of school teaching.

## 2. Marxist Philosophy and System Theory

### 2.1. Marxist Philosophy Course

Philosophy was born from the critical and rational thinking of human beings on life. It is the product of a high degree of spiritual freedom and is a critical and reflective theory. As a branch of philosophy, Marxist philosophy highly develops the essential spirit of philosophy on the basis of practice and is a scientific world outlook and methodology. Based on the essence of Marxist philosophy, realize the optimization of the philosophy education concept from simple, intuitive, abstract, and one-sided to practice, reflection and criticism, people-oriented, and new with the times, so that it can better guide Marxist philosophy education [18].

Marxist philosophy is a science that examines the most fundamental principles guiding the evolution of nature, society, and human thought. It is based on a scientific methodology and worldview. It comes from a variety of particular sciences and is used by particular disciplines. Marxist philosophy has had a significant influence on how human society has evolved, and it continues to be relevant in today's world of constant change by outlining the fundamental guidelines for social development as a whole. Only by making the fundamental ideas of Marxist philosophy clear will it be possible to teach philosophy as philosophy on the basis of understanding the fundamental ideas of philosophy, allowing students to learn the fundamental ideas of Marxist philosophy and solidifying the fundamental ideas of Marxist philosophy position to encourage its development [19]. The characteristics of the essence of Marxist philosophy can still be summed up, despite the fact that from various perspectives, philosophical researchers have different understandings and expressions of the essence of Marxist philosophy.

The Marxist philosophy's usefulness comes first. The most fundamental component of Marxist philosophy is practicality. It permeates the entire theoretical framework from beginning to end as the overarching category of Marxist philosophy. Second is the Marxist philosophy's scientific basis. It has developed into the most thorough and rigorous scientific body unmatched by any other philosophy in the history of human knowledge because it uses the dialectics of materialism as the system's firm foundation and unifies dialectical materialism and historical materialism.

### 2.2. Systems Theory Course

Since Berentaffe's founding, system theory has advanced incredibly quickly, demonstrating not only its robust vitality in the field of application but also the system view and method it has proposed, which have successfully transitioned from experience to philosophy and are now known as system philosophy. According to system theory, the entire world—everything, whether big or small, material or spiritual—exists in a structured manner and is a single organic entity. The world is a systematic place, and the things we deal with can be discussed and studied as a system to discover their inescapable connections, to identify general rules, and to accomplish the goal of comprehending the world and transforming it. Systems theory calls for exactly this. As a result, systems theory is applicable everywhere because it is both a worldview and a methodology. Systems theory has permeated and been broadly adapted in the social sciences as well as the natural sciences, in the organic as well as inorganic, material as well as spiritual worlds. Practice has demonstrated that the systematic worldviews and systematic methodologies advanced by system theory are scientific worldviews and methodologies. It is a high-level generalization and summary of specific sciences and is based on them.

### 2.3. The Connection between Marxist Philosophy and System Theory

Marxist philosophy is a science about the most general rules of the development of nature, society, and human thinking. It is a scientific world outlook and methodology. It originates from various specific sciences and serves specific disciplines. It can be seen that system theory and Marxist philosophy are both scientific world outlook and methodology, and they are at the top of all sciences. In fact, after analyzing and comparing the two, it can be clearly found that system theory and Marxist philosophy are unified with each other, many of their viewpoints are common, and the two can integrate, penetrate, and confirm each other. Many viewpoints of system theory can be reflected from Marxist philosophy, and conversely, many theories of Marxist philosophy can be confirmed from system theory. The two echo each other and complement each other. The point of view on the universal connection and development of things is not only the essence of Marxist philosophy, but also the core content of system theory. So, systems thinking has finally achieved philosophical expression in dialectical materialism.

## 3. Association Rules and Its Application in Course Knowledge Analysis

Association rules, first proposed by Agrawal et al., focus on determining the interrelationships between different attribute domains in the data that meet specific requirements. The association rule mining process is mainly divided into three steps: (1) is to find all frequent item sets that meet the corresponding threshold in the database and gradually find subsets; (2) is to use the mined frequent item sets to generate all the frequent item sets that meet the corresponding threshold, value association rules; and (3) visual processing and evaluation of the discovered rules. The main algorithms used in association rules are Apriori algorithm and its derivatives, incremental mining algorithm, and parallel mining algorithm. The data set analyzed in this paper is small, and the number of iterations is small, so the classic Apriori algorithm is used to perform correlation analysis on courses.

The Apriori algorithm was created and put forth by Agrawal et al. to mine frequently occurring item sets of Boolean association rules. The fundamental concept is to repeatedly scan the database, and its core information is based on the methodical derivation of common item sets. To find the second frequent item set, L2, start by locating the first frequent item set, L1, of the user-defined minsupport threshold. Once no frequent item sets are found, L2 looks for L3, then L3, and so on. Finding frequent item sets is the first step in the implementation process. If an item set is frequent, its subset is also frequent, and the set confidence index determines the rules. Finding rules in the database whose confidence and support are greater than or equal to the specified corresponding thresholds is the main goal of the association rule.

The magnitude of the corresponding probability that the estimated value and the overall parameter are within a certain allowable error range is known as the degree of confidence (abbreviated Dconf) and is another name for confidence. The greater the level of confidence required, the wider the confidence interval will be, reducing the accuracy of the estimate in proportion. Confidence indicates the degree of confidence in the interval estimation. In order to select and determine association rules as a basis for decision-making, you must set your own minimum accuracy value when mining association rules. The formula for calculating the confidence of rules *X* and *Y* is as follows:

(1) $$\begin{array}{c} \text{conf}\left(X⟶Y\right)=\frac{\left|XY\right|}{\left|X\right|}. \end{array}$$

The degree of support is the degree of support (Dsupp for short), that is, the percentage that supports the selected data in a data set. The support formula for item set *X* is

(2) $$\begin{array}{c} D\sup\;p\left(X⟶Y\right)=\frac{\left|X\right|}{\left|D\right|}. \end{array}$$

The formula for calculating the support for rules *X* and *Y* is

(3) $$\begin{array}{c} D\sup\;p\left(X⟶Y\right)=\frac{\left|XY\right|}{\left|Y\right|}. \end{array}$$

The above *X* and *Y* are subsets of the data item set; then, the qualified rule *X* ⟶ *Y* (given the minimum support *α* and the minimum confidence *β*) can be expressed as

(4) $$\begin{array}{c} D\sup\;p\left(X⟶Y\right)\geq \alpha \text{ and }D\text{conf}\left(X-Y\right)\geq \beta . \end{array}$$

There are many studies on the improvement and optimization of association rules and Apriori algorithm in existing literature, and there is few literature applied to curriculum association analysis. A few literature uses student grades or track graduate employment status to obtain data sources to infer curriculum settings. Rationality: This paper takes the Marxist philosophy course as the research object, uses objective data, namely, the course outline to extract content keywords, avoids the influence of other subjective factors, and then uses the Apriori algorithm to extract course association rules to make the analysis results more objective.

## 4. Course Knowledge Association Analysis Model

This paper adopts the Apriori algorithm to analyze the relationship between knowledge. Association analysis is based on the acquired experience value, which comes from the knowledge data obtained after the analysis of students' learning trajectory.  Figure 1 depicts the flow of association analysis of students' course knowledge points.

The steps of students' knowledge correlation analysis are as follows:

(1) From all the learning trajectory data, obtain the student with the largest amount of knowledge, count the knowledge record item set of all students, represent it by knowledge code in the record item set, and record the knowledge record item set as Knowledge_Item.
(2) From the Knowledge_Item data set, traverse each student to find out the knowledge set corresponding to each person, and set the mastered knowledge item set as Point_Item.
(3) Count the frequency value of each knowledge item in the Point_Item in the Knowledge_Item, represented by *C*_*i*_, that is, the frequency value of the *i*-th knowledge item element. The frequency is an absolute value, and the higher the value, the more times this knowledge item appears in the learning analysis.
(4) After calculating the frequency value of each element in Point_Item, calculate the support degree SupportC of each knowledge element.
  (5) $$\begin{array}{c} \text{Support}C_{i}=\frac{B_{i}}{\Delta }\text{Support}C_{i}=\frac{B_{i}}{\Delta }. \end{array}$$
*A* is one of the items in the Knowledge_Item knowledge record item set that pertains to all students in the database, and *B*_*i*_ is the overall number of times the *i*-th knowledge of Point_Item has occurred across all students. If the frequency value is 1, it means that this knowledge occurs when analyzing the knowledge mastery of all students, which indicates whether it is necessary to formulate corresponding knowledge in the learning process of all students. Because the frequency indicates the frequency of a certain knowledge value, if the value is 0, plan for teaching. In light of this, it should be determined whether a given knowledge point is essential knowledge for students if the quantity of samples analyzed reaches a certain threshold (e.g., 200 or more) and the frequency of that knowledge is greater than 0.95. Each student must acquire and master these fundamental skills.
After calculating the support of each knowledge, further calculate the confidence that exists between the two knowledge *C*_*i*_ and *C*_*j*_, as shown in
  (6) $$\begin{array}{c} \text{Confidence }C_{ij}=\frac{Co_{ij}}{B_{i}}. \end{array}$$
In the calculation confidence formula (6), *Co_ij_* is the number of students who have both knowledge of *C*_*i*_ and *C*_*j*_ at the same time, and *B*_*i*_ is the total number of occurrences of the *i*-th knowledge in Point_Item among all students. Confidence *C*_*ij*_ represents the influence of the *i*-th knowledge on the *j*-th knowledge.
(6) In the learning trajectory analysis, set the threshold of the confidence of the association between knowledge, that is, set the threshold to *R*. Generally, this threshold is set according to the actual situation. For example, *R* can be 0.5, 0.6, etc.
(7) Determine the relationship between *R* and confidence *C*_*ij*_. If *R* ≤ confidence *C*_*ij*_, it means that there is an association relationship between the *i*-th knowledge and the *j*-th knowledge in Point_Item, which means that knowledge *C*_i_ is the precondition of knowledge *C*_*j*_. If confidence *C_ij_* = 1, it means that in theory, as long as knowledge *C_i_* appears, knowledge *C*_*j*_ must appear. If confidence *C*_*ij*_ = 0, it means that knowledge *C*_*i*_ and *C*_*j*_ are not related.

In order to determine the relationship between students' mastery of knowledge, it can be represented by a Boolean matrix. In the knowledge-related Boolean matrix model, *M* is the number of rows in the matrix, which is the number of all students to be analyzed, and *N* is the number of columns in the matrix, which is the amount of knowledge mastered by students. Matrix 7 represents the relationship of the number of occurrences between students and knowledge types.

(7) $$\begin{array}{c} D=\left[\begin{array}{ccccccccccc} 0 & 1 & 0 & 1 & 0 & 0 & 0 & 0 & 1 & 0 & 1\\ 0 & 1 & 0 & 0 & 1 & 0 & 0 & 1 & 1 & 1 & 0\\ 0 & 0 & 0 & 0 & 0 & 1 & 0 & 0 & 1 & 1 & 0\\ 1 & 0 & 1 & 0 & 1 & 1 & 0 & 1 & 0 & 0 & 1\\ 1 & 0 & 0 & 1 & 0 & 0 & 0 & 0 & 0 & 0 & 1\\ 1 & 1 & 0 & 0 & 0 & 0 & 1 & 0 & 0 & 0 & 0\\ 0 & 0 & 0 & 0 & 0 & 1 & 0 & 0 & 0 & 1 & 0\\ 1 & 0 & 0 & 0 & 0 & 0 & 0 & 0 & 1 & 0 & 0\\ 1 & 0 & 0 & 0 & 0 & 0 & 0 & 1 & 0 & 1 & 0\\ 0 & 1 & 0 & 0 & 0 & 0 & 0 & 0 & 1 & 0 & 0 \end{array}\right]. \end{array}$$

As shown in matrix 7, in the knowledge matrix, a certain element *D*_*ij*_ of matrix *D* represents the student with the serial number *i*, whether it produces knowledge with the number *j*; if *D_ij_* = 0, it means that the student *i* has no knowledge *j*, and if *D_ij_* = 1, it means that student *i* has knowledge *j*. Through matrix 7, the relationship between knowledge can be easily calculated, including support and confidence.

When the minimum confidence and minimum support are determined one by one, in the generated candidate binomial set, some data are filtered out according to the minimum confidence and support, even if the candidate binomial set between the two knowledge can be further compression. On this basis, focusing on discovering the association rules between knowledge information [20], based on the practical application of the Apriori algorithm, the association analysis of knowledge data is carried out. Through the obtained analysis results, a more scientific learning analysis system can be formulated.

## 5. Correlation Analysis of Curriculum Knowledge

### 5.1. Data Sources

According to the syllabus, the content of the philosophy course is divided into “integrity,” “unity of opposites,” “thing connection,” “practice,” “contradiction,” “dynamic system,” “integrity,” “movement development,” “regular,” and “dialectics.” There are 10 contents in total. Among these knowledge points, “integrity,” “practice,” “movement development,” and “dialectics” belong to the category of Marxist philosophy, while “unity of opposites” and “thing connection” belong to the category of Marxist philosophy, and “dynamic system,” “integrity,” and “rule” belong to the category of system theory.

This paper collects the online test data of 2019 and 2020 students in a university. The test is counted in the above 10 contents, respectively, and the course content score is obtained. That is, first calculate the actual score of each content in the assessment multiplied by the score weight, and sum up to obtain the actual score of the content; then calculate the total score of each content multiplied by the score weight, and sum up to obtain the total score of the content; divide the actual score of the content by the content. The total score and the score data of each course content in [0, 1] can be obtained.

### 5.2. Correlation Analysis of Curriculum Knowledge

Through the analysis of the above data through the Apriori algorithm, valuable course content association rules can be obtained, thus providing help for the improvement of teaching strategies.

The students in this paper are screened out based on their performance on various course assignments. The content that has been chosen is then expressed as an input form that the algorithm can support, and association rules are generated. At the start of the experiment, the experimenter provides the minimum support and minimum confidence. The least frequent of all the recognized item sets, the minimum support degree denotes the lowest statistical importance of the item set. When generating frequent item sets, it is possible to use the minimum support degree to filter out unreliable item sets. Second, choose the low-scoring course material, i. e., the challenging material, in order to generate and analyze the association rules. This is because the level of students' scores is determined by how well they understand the challenging material. After numerous tries, students with content scores below 0.7 were finally eliminated. The support degree was then set to 0.2 when creating frequent item sets, and the minimum confidence degree was then set to 0.45 when creating strong association rules. The result was the 18 items in Table 1.

There are a total of 7 course content items with the support degree greater than 0.15 and the score ratio lower than 0.7, “dynamic system,” “contradiction,” and “wholeness.” Among them, the higher the degree of support, the more the number of people with low scores for the course content item, which is the difficult point that students mastered in teaching. The course content items of “practice,” “unity of opposites,” and “dialectics” did not appear, indicating that students mastered relatively better.

## 6. Analysis of Course Teaching Strategies Based on Association Rules

### 6.1. Key Knowledge Improvement Strategies

1. “Movement development” teaching improvement strategy: the support degree of “movement development” is 44%, which is only lower than 45% of “things connection,” indicating that this is the poor key and difficult content that students have mastered, and it is necessary to focus on analysis and improvement strategies. First analyze the rules 2 and 10 with “motor development” as a precondition; under the premise that “motor development” has a low score, the probability of “integrity” is also low as 58.62%; under the premise that “motor development” has a low score, the possibility of “rule” also scoring low is 64%, both less than 65%, indicating that “movement development” has little effect on other curriculum content.
2. Re-analyzing the rules 1, 7, 8, and 9 of “movement development” as the inferred related content, only the confidence level of rule 8 is 66.66%, which is greater than 65%, which means “contradiction” under the premise that the score is low, “motor development” scores are more likely to be low. In fact, “contradiction” is indeed an important prerequisite for “movement development.” The two have many similar abstract concepts, such as service and protocol characteristics, address classification, and so on. Learning “contradiction” well does have a good guiding effect on the subsequent learning of “motor development.”
3. From the perspective of teaching strategy improvement, teachers can add the internal correlation analysis and comparison between “contradiction” and “movement development” after the teaching of “movement development” to help students master the relationship between the two contents, and appropriately add exercises to consolidate relevant knowledge point, so as to improve the learning effect of students' “motor development.”
4. Teaching improvement strategies of “integrity,” “dynamic system,” and “contradiction”: the support for “integrity” is 33%, the support for “dynamic system” is 32%, and the support for “contradiction” is 23%, all of which are greater than 20%, so “integrity,” “dynamic system,” and “contradiction” can be combined. The content is regarded as the difficulty of the course.
5. First, analyze the rules of these three contents as preconditions. Analyzing the rules 1, 4, 5, and 12 with “integrity” as a precondition, only rule 5 has a confidence greater than 65%. It shows that under the premise of low “integrity” score, the possibility of “contradiction” is also low as 77.27%. Analyzing the rules 3, 7, 13, and 17 with “dynamic system” as a precondition, only rules 3 and 15 have a confidence greater than 65%. Under the premise that the score of “dynamic system” is low, the probability of low score of “integrity” and “contradiction” is 66.66%. Analyzing the rules 6, 8, and 15 with “contradiction” as the precondition, only the rules 6 and 8 have a confidence level greater than 65%. Under the premise that the score of “contradiction” is low, the probability of low score of “integrity” and “motor development” is 66.66%. Then, analyze these three contents as the rules of the inferred related contents, and the rules with a confidence level greater than 65% are also only rules 3, 5, 6, 8, and 13.
6. From the above, it can be seen that the three parts of “integrity,” “dynamic system,” and “contradiction” have a relatively large degree of correlation. In fact, the three are indeed “contradiction” in the “unity of opposites,” and the knowledge points are very high, the degree of correlation. And because these three contents all have certain requirements on students' practical ability, from the perspective of teaching strategy improvement, teachers can appropriately add guidance for these three parts in the teaching process to help students improve “integrity,” “dynamic system,” and the learning effect of “contradiction.”
7. The teaching improvement strategy of “unity of opposites”: The support degree of “unity of opposites” is less than or equal to 0.2, so there are no relevant rules. In fact, this part of the content will be repeatedly mentioned in the teaching content of “unity of opposites” at different levels, and it is more realistic for students to master it relatively well. No changes are needed for the time being.

### 6.2. Unfocused Knowledge Improvement Strategies

1. The teaching improvement strategy of “things connected”: The support degree of the “things connection” course content item is the highest, which is 0.45; that is to say, the number of people with low scores in the “things connection” content learning accounts for 45% of the total number of students, so the “things connection” can be regarded as the hardest content in a part of the course teaching.
2. First analyze the rules of “things connection” as a precondition. Only rule 16 indicates that “things connection” affects the learning of “dynamic system,” but the confidence level is 46.67%, which is less than 65%. In fact, this content has little to do with “dynamic systems.” Reanalyze rules 17 and 18 for “things relation” as inferred relational content. The confidence level is also less than 65%. Therefore, it can be considered that “things connection” is a relatively independent difficult content. This content is at the bottom of the “unity of opposites,” students have less contact in daily life, and the concepts are not easy to understand, so they do have a relatively poor grasp.
3. From the perspective of teaching strategy improvement, since this content is not the focus of the course content, teachers can improve students' learning effect by adding relevant experimental link guidance and exercises.
4. “Regular” teaching improvement strategy: “Regular” support is 38%. Explain that the content of “regular” is relatively poorly grasped by students.
5. Firstly, the rules 9, 11, 14, and 18 with “regular” as preconditions are analyzed, and the confidence levels are not more than 65%. Re-analyzing “regular” as the inferred related content of rules 10, 12, and 15, the confidence level does not exceed 65%. Therefore, it can also be considered that “rule” is a relatively independent difficult content. This content is at the highest level of “unity of opposites” and is closely related to the network activities in life, but the content and classification of the agreement are more, so the students' mastery is relatively poor. From the perspective of teaching strategy improvement, teachers can improve students' learning effect by adding “regular” related exercises and experiments.
6. Teaching improvement strategies of “integrity,” “practice,” and “dialectical”: The support degrees of “integrity,” “practice,” and “dialectical” are all less than or equal to 0.2, indicating that this part of the students has a relatively good grasp, and according to the syllabus, these three parts are all nonkey content. From the perspective of teaching strategy improvement, teachers can appropriately increase online methods to allow students to master these parts more through self-study.

## 7. Conclusions

The association rules of the course teaching material are generated by this paper using the Apriori algorithm based on the key concepts of Marxist philosophy and system theory. It suggests teaching strategies for teachers by examining the association rules between the challenging contents and putting the course syllabus's key points together. The theoretical teaching method for the “movement development” portion of the difficult content could be improved, and link guidance could be added for the “integrity,” “dynamic system,” and “contradiction” portions of the important and difficult content; exercises are added to the “things connection” and “regular” contents; for other parts that are unimportant and straightforward, it is appropriate to direct students through self-study and self-assessment. It is anticipated that the quality of upcoming instruction will improve through the improvement of the aforementioned teaching techniques.

## Figures and Tables

**Figure 1:** Student course knowledge point correlation analysis process.

**Table 1:** Course content difficulties in strong association rules.

Serial number	Strong association rules	Dsupp	Dconf
1	“Integrity” ⟶ “movement development”	0.33	0.4545
2	“Movement development” ⟶ “integrity”	0.44	0.6666
3	“Dynamic system” ⟶ “integrity”	0.32	0.4545
4	“Integrity” ⟶ “dynamic system”	0.33	0.7727
5	“Integrity” ⟶ “contradiction”	0.33	0.6666
6	“Contradiction” ⟶ “wholeness”	0.23	0.5238
7	“Dynamic systems” ⟶ “motion development”	0.32	0.6666
8	“Contradiction” ⟶ “movement development”	0.23	0.5600
9	“Rule” ⟶ “movement development”	0.38	0.6400
10	“Movement development” ⟶ “regulations”	0.44.	0.5200
11	“Rule” ⟶ “integrity”	0.38.	0.5909
12	“Integrity” ⟶ “rule”	0.33	0.6666
13	“Dynamic system” ⟶ “contradiction”	0.32	0.5517
14	“Rule” ⟶ “dynamic system”	0.23	0.4762
15	“Contradiction” ⟶ “rule”	0.45.	0.4667
16	“Thing connection” ⟶ “dynamic system”	0.32	0.4545
17	“Dynamic system” ⟶ “thing links”	0.38	0.5200
18	“Rule” ⟶ “thing connection”	0.33	0.4545

## Data Availability

The data used to support the findings of this study are available from the corresponding author upon request.
